This article has been retracted.

# Analysis and Study on the Quality of Life of Patients Undergoing Transcatheter Aortic Valve Replacement

**DOI:** 10.1155/2021/3147382

**Published:** 2021-12-16

**Authors:** Guoliang Wu, Jiajun Zhu, Kaixuan Hu, Huan Cai, Xiaomei Li, Yining Yang

**Affiliations:** ^1^Department of Cardiology, The First Affiliated Hospital of Xinjiang Medical University, Urumqi, 830001 Xinjiang, China; ^2^Department of Cardiology, People's Hospital of Xinjiang Uygur Autonomous Region, Urumqi, 830001 Xinjiang, China

## Abstract

**Objective:**

Explore the factors affecting the QO of life after transcatheter aortic valve replacement (TAVR) and analyze and evaluate their surgical efficacy and postoperative survival status.

**Methods:**

Through correlation analysis and multiple regression analysis, we predict various clinical characteristics and postoperative quality and predict clinical changes in L postoperative quality.

**Results:**

The quality of life of patients with the disease has gradually improved and improved from 6 months after surgery. The differences in the three aspects of its physiological mechanism function, physiological function function, overall health, and vitality are statistically significant (*p* < 0.05).

**Conclusion:**

Compared with traditional open-thoracic aortic valve (AV) surgery, TAVR has the significant advantages of smaller surgical incision and less trauma to the patient, which has become one of the reasons why patients are willing to accept it.

## 1. Introduction

With the development of the aging population, elderly degenerative heart disease becomes more and more common, and aortic valve stenosis (aorticstenosis, AS) has become one of the common heart diseases following coronary heart disease, hypertension, and once clinical symptoms appear, the fatality rate of 50%~75%. As the average age of the Chinese population continues to rise, the prevalence of some diseases is also rising. Investigations and studies on the elderly have shown that heart disease, especially aortic stenosis(AS), poses a major threat to human health [1, 2]. With the development of catheter technology, fewer complications and better availability mean that more patients will consider AV replacement. TAVR has become an intolerable operation and the main treatment method and means for patients with chronic AS with high-risk surgical characteristics and indications [3, 4].

At present, many domestic and foreign scholars have conducted research on AV stenosis and its treatment methods and have achieved good results. Some scholars have shown that TAVR has expanded the treatment field of high-risk patients with AV stenosis. The results show that TAVR is feasible and is a high-risk or severe symptomatic subject with surgical contraindications. Patients with valvular stenosis provide midterm hemodynamics and clinical improvement [5]; TAVR has been shown to significantly improve patients with severe AS who cannot perform surgical cardiovascular disease surgery as compared to standard treatment. Studies by some scholars have shown that the TAVR trials randomized severe AS patients not suitable for surgical valve replacement for cardiovascular disease to TAVR (*n* = 179) or standard therapy. The Kansas City Cardiomyopathy Questionnaire (KCCQ) and the 12-item 12 Comprehensive Health Survey (SF-12) were used to assess health-related quality of life at baseline and 1, 6, and 12 months [6]. Other researchers have also shown that TAVR using the sapien 3 valve has shown good 30-day clinical results in patients with severe AS at a moderate risk of surgical death. They reported receiving SAPIEN 3 TAVR long-term data of intermediate-risk patients, and the results were compared with those of intermediate-risk patients undergoing surgical AV replacement [7]. In addition, researchers are trying to evaluate the potential definition of adverse outcomes after TAVR combined with mortality and life treatments. Using data from a subset of 463 patients who underwent TAVR surgery, they evaluated their 6-month mortality and life. For quality results, use the KCCQ to explore potential definitions of adverse outcomes, and finally, compare the advantages and disadvantages of each potential definition by examining the relationship between them [8]. In conclusion, the results of the current studies on atrioventricular stenosis and its treatment are very mature and provide a theoretical basis for the study in this paper.

The analysis of treatment for atrioventricular stenosis, TAVR complications, and TAVR adaptation population was selected from July 2012 to July 2020. For patients undergoing valve replacement, a three-dimensional analysis of postoperative quality of life was performed, because the scope and data involved were more accurate, so a 3-dimensional method (the SF-36 health survey questionnaire) was selected for postoperative quality analysis. Patients were assessed using a quality of life scale score and found a significant improvement in the upper half of surgery compared with the baseline survey.

## 2. Analysis and Study on the Quality of Life of Patients Undergoing TAVR

### 2.1. The Treatment of AS

1. Surgical treatment

For adult patients with severe AS, surgery is a level I recommendation in the heart valve guidelines. The doctor's experience and the continuous improvement of valve technology have significantly improved the surgical method, the success rate of surgical treatment, and the long-term survival rate (SR) after surgery. For some adult patients with severe symptoms, surgical treatment is effective and safe [9]. However, about one-third of patients tend to suffer from multiple diseases, and their general health is not suitable for surgical treatment. Therefore, surgical treatment is not applicable to all adult patients with severe AS symptoms, especially in elderly patients who often have multiple comorbidities.

(2) Percutaneous balloon aortic valvuloplasty

Percutaneous balloon aortic valvuloplasty is the oldest method used to treat AS through a catheter. This kind of drug treatment can only effectively improve patient's blood flow and relieve the symptoms in a short period of time. About 80% of cases will relapse within 6-12 months after surgery and cannot improve their SR. Generally speaking, it is only used as a surgical method for surgical treatment and AV replacement through catheters that have contraindications or other transitional treatments [10].

(3) TAVR

Medications and PBAV were not effective in adult patients with severe AS symptoms. SAVR is an effective tool to alleviate clinical symptoms in patients with high-risk surgery and improve long-term survival, postoperative mortality, and side effects. However, patients with high risk of surgery had very high postoperative mortality and adverse events. With that in mind, cardiologists need to find new technology. The TAVR procedure is shown in Figure 1.

(4) Drug treatment

Patients with AS who cannot undergo surgery require long-term medication. Since hypertension is an important risk factor for AS, patients with AS should receive standard antihypertensive treatment. Vasodilators can be used in patients with severe compensatory heart failure. However, drug therapy can only target coexisting cardiovascular diseases or slow the progression of AS. Patients with slow-growing AS may experience worsening symptoms and repeated hospitalizations even if they are given the best medications. There is currently no evidence that drug therapy can effectively improve survival [11].

### 2.2. Complications of TAVR

1. Artificial AV regurgitation

Artificial aortic regurgitation is a common condition after TAVR, and there is no significant difference in the incidence of self-expanding valves and balloon-expanding valves. The evaluation of reflux shall be divided into two parts: beside valve leakage and inside valve reflux. The current guidelines use echocardiography to quantitatively and semiquantitatively evaluate hemodynamics, paravalvular leakage at the lower end of the prosthetic valve stent, and the degree of regurgitation at the junction of the prosthetic valve leaflets and evaluate the intravalvular regurgitation at the prosthetic leaflet junction degree. In addition, X-ray photography of the aortic root is also a practical and effective method to evaluate aortic regurgitation. Usually, the function of the implant valve can be evaluated after TAVR.

(2) Stroke

The clinical nature of acute stroke after TAVR is basically considered to be ischemic stroke. The main pathological cause may be the appearance of ruptured small holes in the blood vessel wall and the cerebral valve itself, which causes cerebral vascular embolism. One of the main causes of subacute stroke is the formation of thrombus, which is mainly related to the artificial valve leaflet damage caused by the exposure of the artificial valve leaflet stent, valve preinstallation and balloon expansion, and the exposure of the artificial valve leaflet stent after injury. Platelets and fibrin aggregates are associated with unique valves [12].

(3) Paravalvular leak

Paravalvular leak is a common complication after TAVR. Studies have shown that mild paravalvular leakage has no significant effect on the prognosis of patients, and only moderate to severe paravalvular leakage is associated with patient mortality. The chamber ring is a noncircular three-dimensional structure. It is very important to accurately measure the relative diameter of the atrial chamber ring before the TAVR. Incomplete extension of the artificial scaffold frame or incorrect valve implantation location is related to the occurrence of paravalvular leakage.

(4) Stroke

Stroke is a common and important complication of TAVR, mainly including stroke and transient ischemic attack. Most of them are related to the rejection of intraoperative aortic membrane calcification or aortic arch sclerosis plaque, and the incidence rate within 30 days after surgery is 1% to 11%. Strokes mainly occur in the early stages after TAVR, approximately 25% to 50% occur within 24 hours after surgery, and 80% occur within 5 days after surgery. Asymptomatic microembolism after TAVR can affect the cognitive function of patients and cause dementia. On the other hand, stroke will increase the mortality of patients and affect the self-care ability and quality of life of patients after surgery.

### 2.3. TAVR Is Adapted to the Crowd

1. Patients with low surgical risk

Since the launch of TAVR, clinical trials have continuously evaluated its effectiveness and safety. According to different risk stratification, it can be divided into four categories: surgical contraindications or extremely high-risk, high-risk, and medium-low-risk. The 2014 ESC/EACTS valvular disease guidelines recommend TAVR for severe symptomatic AS, STS score > 10%, or EuroSCORE ≥ 20%. Currently, only TAVR is recommended as an alternative to surgical contraindications. For patients with a high risk of surgery that may undergo SAVR, treatment and TAVR are not recommended as class I recommendations.

(2) Patients with bicuspid AS

TAVR is still in its infancy in China. Chinese patients with AV stenosis have severe AV leaflet and annular calcification, and the incidence of AV malformation is high. However, most large randomized controlled trials abroad have excluded bicuspid valves, clinical BAV, and TAV after AV replacement. A meta-analysis has compared the effects: there were no statistically significant differences in postoperative in-hospital mortality, 30-day mortality, and 1-year mortality between the two groups. The surgical success rate, postoperative bleeding event, and postoperative vascular injury were lower than BAV and were statistically significant.

(3) Patients with simple aortic regurgitation

TAVR treatment has the advantages of less trauma and quick recovery. Clinical studies have shown that TAVR is a simple aortic regurgitation, because some patients with aortic regurgitation cannot tolerate surgery and receive appropriate treatment. Whether it can be applied is under study. Since a key condition for the application of TAVR is the calcification of the natural valve, the calcified natural valve imparts radial bearing capacity to the embedded prosthesis and forms a fixed anchor. Patients with simple aortic insufficiency have less valve calcification, so TAVR is more difficult to perform than patients with AS, and the risk of moderate to severe paravalvular leakage is increased.

## 3. Experiment

### 3.1. Case Selection Criteria

This article selects 108 patients undergoing AV replacement in a hospital from July 2012 to July 2020 (a publicly available data resource), including 58 males and 50 females, with an average age of 52.68 ± 13.42 years old. Patients over 60 years old account 36.8% for the total number of patients. Inclusion criteria: (1) patients who are not treated before surgery or have no diabetes, cerebrovascular, and other diseases that may affect their health and quality of life; (2) patients who can voluntarily sign up for this research work and have a considerable degree of compliance.

### 3.2. Exclusion Criteria

1. Patients who cannot be followed up after surgery
2. Patients with other diseases that affect the quality of life

### 3.3. Statistical Processing

This article uses SPSS24.0 for statistical data analysis and GraphPrism7.0 for drawing. The data is divided into continuous variables and categorical variables according to their characteristics. You need to check the regularity of continuous variables. Continuous variables that match the normal distribution are expressed as mean ± standard deviation. The independent sample *t*-test is used to compare the differences between the two groups. Categorical variables are expressed as frequencies (percentages), and use a chi-square test to compare the differences between the two groups. If necessary, choose continuity correction (1 < *T* < 5) or exact Fisher's exact test (*T* < 1) based on the expected frequency *T* results. All data use a bilateral test. If *p* < 0.05, it is considered statistically significant. The test statistics are:

(1) $$\begin{array}{c} t=\frac{\bar{X}-\mu }{\sigma_{X}/\sqrt{n-1}}. \end{array}$$

If the sample is a large sample, it can also be written as:

(2) $$\begin{array}{c} t=\frac{\bar{X}-\mu }{\sigma_{X}/\sqrt{n}}. \end{array}$$

Here, $\bar{X}$ is the sample average, *μ* is the overall average, *σ*_*X*_ is the sample standard deviation, and *n* is the sample size.

## 4. Discussion

### 4.1. Replacement of Different Types and Models of Artificial Active Valve EOA Reference Value

As can be seen from Table 1 and Figure 2, there are 24 patients with mechanical replacement valve St. Jude, 3 patients with mechanical valve replacement St. Jude Regent, 19 patients with mechanical valve replacement ATS, and 38 patients with mechanical valve replacement Carbomedics; there were 16 patients with Hancock II replacement biovalves, 8 patients with CE Porcine replacement biovalves; 84 patients replaced mechanical valves, and 24 patients replaced biovalves.

### 4.2. Comparison of SRs between Matched Group and Unmatched Group of Artificial Valve Patients

It can be seen from Table 2 that the SR of patients with mild prosthetic valve mismatch after six months was 42.5%, the SR of patients with moderate mismatch was 29.5% after six months, and the SR of patients with severe mismatch was 29.5% after six months. The SR of patients with mild prosthetic valve mismatch was 41.6% after 1 year, the SR of patients with moderate mismatch was 27.1% after 1 year, and the SR of patients with severe mismatch was 27.1% after 1 year. 26.1%; the SR of patients with mild prosthetic valve mismatch was 40.3% after 3 years, the SR of patients with moderate mismatch was 25.7% after 3 years, and the SR of patients with severe mismatch was 23.6 after 3 years %; the SR of patients with mild prosthetic valve mismatch after 5 years is 40.3%, the SR of patients with moderate mismatch is 21.3% after 5 years, and the SR of patients with severe mismatch is 19.2% after 5 years; the SR of patients with mild prosthetic valve mismatch after 7 years was 37.2%, the SR of patients with moderate mismatch was 16.6% after 7 years, and the SR of patients with severe mismatch was 12.7% after 7 years.

As shown in Figure 3, SR for artificial valve mismatch was 100%, 94.8%, and 89.6% after 1 year, 66.5% after 5 years and 1 year, 90.9% after 3 years, 84.3% after 5 years, and 77.4% after 7 years. Overall, patients with matched artificial valves had significantly higher SRs than those with an artificial valve mismatch.

### 4.3. Comparison of Postoperative Quality of Life

According to Table 3 and Figure 4, through a comprehensive assessment of the scores of the quality of life evaluation indicators, it is found that the patients with this disease have significantly improved their quality of life after investigation on a relative baseline within half a year after surgery. The scores of the time period were higher than those before the operation, and the differences in the four aspects of physiological mechanism, physiological intelligence, overall health, and vitality were statistically significant (*p* < 0.05).

## 5. Conclusions

TAVR expands the field of treatment in patients at high risk for AV stenosis. The results suggest that TAVR is feasible and a surgical contraindication for high-risk or severe symptoms. Patients with valve stenosis can provide midterm hemodynamic and clinical improvement.

At present, as TAVR continues, indications expand to young and low-risk patients. Meanwhile, some current experimental data also provide the possibility of applying TAVR to lobular and aortic regression. Increasingly, clinicians have reported postoperative complications of TAVR. At present, we believe that complications after TAVR can be well addressed by in-depth research, valve development, and technical improvements.

## Figures and Tables

**Figure 1:** TAVR surgery flow chart.

**Figure 2:** Number of cases of different valve types.

**Figure 3:** Comparison of SRs between matched group and unmatched group of prosthetic valve patients (%).

**Figure 4:** Comparison of scores in various dimensions with baseline surveys in the first half of the postoperative period.

**Table 1:** Replacement of different types and models of artificial active valve EOA reference value.

Valve type		Artificial valve model (mm) and effective opening area (cm^2^)				
		19	21	23	25	27
Mechanical flap	St. Jude	1.03	1.37	1.51	2.07	2.64
	St. Jude Regent	1.69	2.99	2.39	2.49	3.59
	ATS	1.19	1.49	1.74	2.14	2.50
	Carbomedics	1.00	1.53	1.62	1.97	2.40

Bioprosthesis	Hancock II	None	1.17	1.32	1.45	1.54
	CE Porcine	1.05	1.39	1.45	1.51	1.87

**Table 2:** Comparison of SRs between matched group and unmatched group of prosthetic valve patients (%).

Unmatched group					Matching group
Time/y	Mild	Moderate	Severe	Total	Total
0.5	42.5	29.5	28	100	100
1	41.6	27.1	26.1	94.8	93.9
3	40.3	25.7	23.6	89.6	90.6
5	40.3	21.3	19.2	80.8	84.3
≥7	37.2	16.6	12.7	66.5	77.4

**Table 3:** Comparison of scores in various dimensions with baseline surveys in the first half of the postoperative period.

Item	Before surgery	Postoperative	t value	p value
Physiological function	63.93±7.35	68.97±8.23	3.323	0.001
Body pain	67.15±10.63	69.86±9.13	1.493	0.067
General health	37.58±11.76	44.14±12.33	2.751	0.006
Vitality	56.79±8.09	61.19±7.41	2.918	0.003
Social function	58.62±7.60	60.15±8.11	1.124	0.080
Affective function	63.56±8.60	64.81±7.42	0.427	0.652
Mental health	68.03±9.49	69.00±9.03	0.983	0.120

## Data Availability

The data underlying the results presented in the study are available within the manuscript.
